# A Neighborhood Model with Both Distance and Quantity Constraints for Multilabel Data

**DOI:** 10.1155/2022/9891971

**Published:** 2022-09-19

**Authors:** Xiaoli Jiang, Jing Zhou, Xinyue Qiao, Chang Peng, Shiwen Su

**Affiliations:** College of Mathematical Sciences, Bohai University, Jinzhou 121013, China

## Abstract

In this paper, a novel distance-based multilabel classification algorithm is proposed. The proposed algorithm combines k-nearest neighbors (kNN) with neighborhood classifier (NC) to impose double constraints on the quantity and distance of the neighbors. In short, the radius constraint is introduced in the kNN model to improve the classification accuracy, and the quantity constraint *k* is added in the NC model to speed up computing. From the neighbors with the double constraints, the probabilities for each label are estimated by the Bayesian rule, and the classification judgment is made according to the probabilities. Experimental results show that the proposed algorithm has slight advantages over similar algorithms in calculation speed and classification accuracy.

## 1. Introduction

The multilabel classification problem stems from the text and image classification [1]. In practice, a text often has multiple keywords, and an image often has multiple scenes [2]. The authors of [3] proposed a multi-instance multilabel learning (MIML) approach for large datasets via subspace technique and stochastic gradient descent. To handle a data stream, an approach called multilabel learning with emerging new labels (MuENL) was proposed [4]. Combining the mixed dependency graph and the class cooccurrence, the authors of [5] constructed an optimization problem to deal with the label relevance for the multilabel learning with missing labels (MLML) and applies the ADMM algorithm to solve it. In reference [6], Zhang et al. reviewed the problem of binary correlation in multilabel learning.

The multilabel classification can be converted into a single-label problem by treating the labels as the vector value. However, the computational complexity is intolerable. In order to improve the computational speed, an improved algorithm called random k labelsets (RAkEL) was proposed [7]. Zhang and Zhou [8] established a multilabel version of kNN by Bayesian rule, and named it multilabel k-nearest neighbors (ML-kNN). In their experiments, ML-kNN was compared with the multilabel classification algorithms BOOSTEXTER [9], ADTBOOST.MH [10], and RANK-SVM [11]. ML-kNN treats each label as an independent binary classification and ignores the correlation between the labels. In order to make use of the correlation between the labels, the authors of [12] regarded the neighbor's labels as the features of instances and gave an extension of ML-kNN. For multilabel data streams, self-adjusting memory (SAM) [13] was adopted to deal with data drifting, and a multi-label k-nearest neighbor (ML-SAM-kNN) was established [14].

As well known, the kNN algorithm makes prediction by investigating the k-nearest neighbors of the unknown instances. Each instance is assigned a uniform parameter k. This is based on the assumption that the data is evenly distributed. In reality, most data are not uniformly distributed. The certainty factor measure [15] was designed for kNN classification to deal with to the skewed class distribution. Meanwhile, the shell neighbor imputation [16] fills the incomplete data by left and right nearest neighbors. For noisy data, the pseudo-nearest neighbors was identified by mutual k-nearest neighbor [17].

For a long time, the choice of parameter k was empirical. For example, the authors of [18] have tried to take it as the square root of the sample size, which does not address the problem of the uneven data. In view of this, the method of selecting different parameter k for different samples was proposed [19]. Different k values were learned by correlation matrices and assigned to different test data points [20]. A kTree method [21] to learn different optimal k values for different test samples was proposed with a sparse reconstruction model. The cost-sensitive kNN classifiers were designed and further improved with minimum-cost k-value selection, feature selection, and ensemble selection [22]. However, it will greatly increase the complexity of the kNN model and reduce the robustness of the algorithm. In extreme cases, if the different parameter is set for each sample, the computational complexity is unacceptable, especially for large data. In the [23], large data were first separated into several parts by k-means clustering, each of which has then conducted the kNN classification.

The kNN is a distance-based classifier, which estimates the labels of unknown instances according to the labels of the nearest neighbors. Therefore, the distance between the nearest neighbor and the unknown instance has a great impact on the accuracy of the estimation. In fact, with the increase of the distance from the unknown instance, the reference value of the nearest neighbors decreases gradually. In [24], a distance-weighted k-nearest neighbor algorithm (DW-kNNA) was introduced to solve a permanent magnet synchronous linear motor (PMSLM) model. Alfeilat, Hassanat, Lasassmeh, et al. showed that the performance of kNN classifier depends significantly on the distance used [25]. The *l*_21_-norm based distance measurement was adopted in the loss function to improve the model robustness [26]. Meanwhile, the mathematical framework based on differential evolution with compressed sensing can learn the sparse module dictionaries and levels from the low-dimensional random composite measurements for reconstructing the high-dimensional data [27]. In 2020, a locality-constrained graph was introduced in the nonnegative matrix factorization algorithm to discover the geometric structure of the data [28]. A novel machine learning method based on the modified kNN algorithm was proposed. More features can be extracted from the datasets, and the datasets were updated during the training process instead of constructing the dataset beforehand [29], where a computational framework based on compressed sensing can be adopted to reduce dimensionality [30].

However, when the distance between the training instance and the unknown instance exceeds a certain value, the information of the nearest neighbors not only has no reference value for the judgment of the unknown instance, but also sometimes leads to misleading.  Figure 1 shows a binary classification problem with nonuniformly distributed data. Assuming that the problem is linearly separable, the straight lines in the figure represents the classification hyperplane. The question mark “?” is an unknown instance, as shown in Figure 1(a), whose 3NN contains two positive instances and one negative instance. However, the correct judgment is that the unknown instance belongs to the negative class. The distance range investigated by the algorithm 3NN is too large in the sparse area. When the training instances are far away from the unknown instances, it means that their features are quite different from those of the unknown instances. At this point, it is easy to get wrong estimates if these training instances are considered as the classification basis. In view of the above analysis, we can assume that the referential meaning of the training instance is lost when its distance from the unknown instance exceeds a certain value. In other words, we just take the training instance within a certain range centered the unknown instance as classification basis.

Based on the above assumptions, we append a new parameter in the kNN model, which is the distance centered on an unknown instance. Only the *k*-nearest neighbors whose distance from the unknown instance is less than the given value are utilized for prediction. The neighbors for prediction are constrained by both quantity and distance. The distant constraint aims to pick up a certain number of neighbors among the *k*-nearest neighbors. As shown in Figure 1(b), the label of the unknown instance can be correctly judged by the nearest neighbor with the distance constraint. At this point, the two positive instances in 3 nearest neighbors will no longer be used as reference.

In the neighborhood classifier, the neighborhood contains a large number of instances for the data with high distribution density, especially numerical data. The computation complexity will be greatly increased by counting the label information of the neighbors in the neighborhood. In order to improve the computational efficiency, we only consider the k-nearest neighbors in the neighborhood as the reference for classification.

Different from simple label classification and the classification based on density estimation, multilabel classification predicts a set of labels associated with each sample, where the number and category of labels are both random. Therefore, the complexity of multilabel classification is exponentially higher than that of unilabel classification and the classification based on density estimation, which is also one of the main problems faced by multilabel classification. In order to alleviate the exponential growth, multilabel classification tasks are decomposed into independent single-label classification tasks in this paper. It not only reduces the complexity of the problem, but also facilitates parallel computing.

In Section 2, we present a mathematical description of the multilabel classification and introduce some of the symbols and concepts to be used. A novel multilabel classification algorithm based on ML-kNN and the neighborhood classifier will be presented in Section 3. In order to verify the effectiveness of the algorithm, we selected some common multilabel data and carried out some comparative experiments. The results will be reported and analyzed in Section 4.

## 2. Preliminaries

Multilabel training data are composed of features and labels. The features are measurable properties of an instance. The labels represent the classes to which the instance belongs. The purpose of classification learning is to train a classifier from the feature and label data. The classifier can predict the class labels from the measurable features.

Let *X* be a nonempty finite set of instances. An instance can be denoted as a vector *x*=(*x*_1_, *x*_2_,…, *x*_*n*_) ∈ *X*, which implies that its feature values are *x*_1_, *x*_2_,…, *x*_*n*_, respectively. The numerical and nominal feature values are expressed as real numbers and natural numbers, respectively. The distance between the instances is defined as

(1) $$\begin{array}{c} d\left(x,x^{\prime }\right)=\sqrt{\overset{n}{\underset{i=1}{\sum }}d_{i\left(x_{i},x_{i}^{\prime }\right)}},x,x^{\prime }\in X\text{.} \end{array}$$

For numeric features, let

(2) $$\begin{array}{c} d_{i}\left(x_{i},x_{i}^{\prime }\right)={\left(x_{i}-x_{i}^{\prime }\right)}^{2}\text{,}\\ d_{i}\left(x_{i},x_{i}^{\prime }\right)=\left\{\begin{array}{cc} 1\text{,} & x_{i}=x_{i}^{\prime }\text{,}\\ 0\text{,} & x_{i}\neq x_{i}^{\prime }\text{,} \end{array}\right.,x,x^{\prime }\in X\text{,} \end{array}$$

be nominal features. For each instance *x* ∈ *X*, let *N*^*k*^(*x*) denote the set of kNNs of *x*, and the set *N*_*δ*_(*x*)={*y* ∈ *X* : 0 < *d*(*x*, *y*) ≤ *δ*} is said to be the *δ*-neighborhood of the instance *x*. The elements in the intersection

(3) $$\begin{array}{c} N_{\delta }^{k}\left(x\right)=N_{\delta }\left(x\right)\cap N^{k}\left(x\right)\text{,} \end{array}$$

are called *δ*-kNNs of the instance *x*.

Let *L* be the collection of labels. The multilabel classification is to learn a function *h* : *X*⟶2^*L*^ from the training data

(4) $$\begin{array}{c} D=\left\{\left(x,L_{x}\right):x\in X\right\}\text{,} \end{array}$$

where the label subset *L*_*x*_ ⊂ *L* is the set of labels associated with the instance *x*. Each label *l* ∈ *L* defines a random variable *l* : *X*⟶{0,1}. If the instance *x* has the label *l* ∈ *L*, then *l*(*x*)=1, otherwise, *l*(*x*)=0. A random variable *C*^*k*^ : *X*⟶{0,1,…, *k*} is defined as

(5) $$\begin{array}{c} C^{k}\left(x\right)=\underset{x^{\prime }\in N^{k}\left(x\right)}{\sum }l\left(x^{\prime }\right),\forall x\in X\text{,} \end{array}$$

to count the number of the instances with the label *l* ∈ *L* in the neighborhood *N*^*k*^(*x*). In the same way, a random variable *C*_*δ*_ : *X*⟶*Z*^+^ is defined as

(6) $$\begin{array}{c} C^{k}\left(x\right)=\underset{x^{\prime }\in N_{\delta }\left(x\right)}{\sum }l\left(x^{\prime }\right),\forall x\in X\text{,} \end{array}$$

to count the number of the instances with the label *l* ∈ *L* in the neighborhood *N*_*δ*_(*x*), where *Z*^+^ is the positive integer set.

Multilabel k-nearest neighbor (ML-kNN) makes prediction with the label information embodied in the k neighbors by the maximum a posteriori (MAP) rule. The pseudo-code of ML-kNN is shown in Table 1. Here, we only listed the basic framework to illustrate its idea, see [1, 8] for details.

The innovation of this paper lies in the establishment of a new algorithm combining the ideas of ML-kNN and neighborhood classifier (NC) [31]. The pseudo-code of NC is given in Table 2 to illustrate the basic idea of the proposed algorithm.

From Table 1 and Table 2, it can be seen that the difference between the two algorithms lies in the definitions of the neighborhoods. The algorithm ML-kNN limits the number of the neighbors, while NC restricts the distance of neighbors. The proposed algorithm in this paper will double constrain the nearest neighbor from both quantity and distance.

## 3. Bounded ML-kNN

In order to reduce the computational burden, a new radius parameter is introduced into the kNN model to reduce the number of neighbors, and a novel mult-label classification algorithm is established in this section.

We decompose the multilabel data *D* into a series of binary classification data.

(7) $$\begin{array}{c} D_{l}=\left\{\left(x,l\right):x\in X\right\},l\in L\text{,} \end{array}$$

which are single-label data with the same feature data as the multilabel one *D*. Then, the classifier deals with each binary classification independently. The neighborhood *N*_*δ*_^*k*^(*x*) of each instance *x* ∈ *X* is calculated according to the distance defined in Section 2. The random variables *C* : *X*⟶{0,1,…, *k*} can be defined as

(8) $$\begin{array}{c} C\left(x\right)=\underset{x^{\prime }\in N_{\delta }^{k}\left(x\right)}{\sum }l\left(x^{\prime }\right),\forall x\in X\text{,} \end{array}$$

to count the number of the instances with the label *l* ∈ *L* in the neighborhood *N*_*δ*_^*k*^(*x*). The label *l* of each instance *x* ∈ *X* is estimated by maximizing the posteriori probability *p*(*l*|*C*), i.e.,

(9) $$\begin{array}{c} l\left(x\right)=arg\;\max_{l\in \left\{0,1\right\}}\;p\left(\left.l\right|C\left(x\right)\right)\text{,} \end{array}$$

where the symbol *C*(*x*) represents the random event *C*=*C*(*x*) that there are *C*(*x*) instances with the label *l* in the neighborhood *N*_*δ*_^**k**^(*x*) of the instance *x* ∈ *X*. The number *C*(*x*) could be any positive integer between 0 and *k*. Bayes' theorem implies

(10) $$\begin{array}{c} p\left(\left.l\right|C\right)=\frac{p\left(l\right)p\left(\left.C\right|l\right)}{p\left(C\right)}\text{.} \end{array}$$

Since *p*(*C*) is constant whether *l*=1 or *l*=0, the optimization problem can be reduced to

(11) $$\begin{array}{c} l\left(x\right)=arg\;\max_{l\in \left\{0,1\right\}}\;p\left(l\right)p\left(\left.C\left(x\right)\right|l\right)\text{.} \end{array}$$

In the training phase, we learn the probability *p*(*l*) from the training data *D*_*l*_. The symbol |*X*| represents the cardinality of the set *X*, i.e., the total number of instances in the set *X*. The ratio

(12) $$\begin{array}{c} \frac{\sum_{x\in X}l\left(x\right)}{\left|X\right|}\text{,} \end{array}$$

is taken as an estimate of the probability *p*(*l*=1). For the convenience of computer calculation, we introduce an auxiliary parameter *s*, so that the probabilities can be approximated as

(13) $$\begin{array}{c} p\left(l=1\right)=\frac{s+\sum_{x\in X}l\left(x\right)}{2s+\left|X\right|}\text{,} \end{array}$$

(14) $$\begin{array}{c} p\left(l=0\right)=1-p\left(l=1\right)\text{.} \end{array}$$

The second probability to be learned is the conditional probability *p*(*C*|*l*). Consider the following instance sets

(15) $$\begin{array}{c} D_{j}^{1}=\left\{x\in X:C\left(x\right)=j,l\left(x\right)=1\right\},j=0,1,\ldots ,k\text{,}\\ D_{j}^{0}=\left\{x\in X:C\left(x\right)=j,l\left(x\right)=0\right\},j=0,1,\ldots ,k\text{,} \end{array}$$

which are the sets of the training instances *x* with the label *l* (when *l*(*x*)=1) or without the label *l* (when *l*(*x*)=0), while each *x*'s neighborhood *N*_*δ*_^**k**^(*x*) contains exactly *j* neighbors with the label *l*. Therefore, the conditional probabilities *p*(*C*=*j*|*l*=1) can be approximated by the ratio

(16) $$\begin{array}{c} \frac{\left|D_{j}^{1}\right|}{\sum_{j=0}^{k}\left|D_{j}^{1}\right|}\text{,} \end{array}$$

where the cardinality of the set *D*_*j*_^1^ is denoted by |*D*_*j*_^1^|, which is equal to the number of the instances in the set *D*_*j*_^1^. The auxiliary parameter *s* is introduced to establish the estimation

(17) $$\begin{array}{c} p\left(\left.C=j\right|l=1\right)=\frac{s+\left|D_{j}^{1}\right|}{s\left(k+1\right)+\sum_{j=0}^{k}\left|D_{j}^{1}\right|}\text{.} \end{array}$$

Similarly, we can obtain the estimation

(18) $$\begin{array}{c} p\left(\left.C=j\right|l=0\right)=\frac{s+\left|D_{j}^{0}\right|}{s\left(k+1\right)+\sum_{j=0}^{k}\left|D_{j}^{0}\right|}\text{.} \end{array}$$

For each unknown instance *t*, the label is determined by the following principle:

(19) $$\begin{array}{c} l\left(t\right)=arg\;\max_{l\in \left\{0,1\right\}}\;p\left(l\right)p\left(\left.C\left(t\right)\right|l\right)\text{.} \end{array}$$

The pseudo-code for bounded ML-kNN (BML-kNN) is presented in Table 3.

In the pseudo-code, the multilabel classification is decomposed into the independent single-label problem for each label *l* ∈ *L*. From Step 2 to Step 16, the probabilities *p*(*l*) and *p*(*C*|*l*) are learned from the single-label training data. The counter *c*(*j*) records the number of the training instances with the label *l*, and whose neighborhood contains *j* instances with the label *l* for each *j*=0,1,2 · , *k*. Simultaneously, the counter $\bar{c}\left(j\right)$ is the total number of training instances without the label *l*, and whose neighborhood contains *j* instances with the label *l*. From Step 17 to Step 20, the optimization problem can be solved by applying the probabilities (13), (14), (17), and (18). The labels of the unknown instances are given one-by-one.

## 4. Experiment Results

In this section, some experimental results are reported to compare our proposed methods with ML-kNN. The experiments were conducted on a computer with Intel(R) Core(TM) i5-7200U CPU at 2.50 GHz and 16 GB memory. Some common and typical multilabel datasets were selected as experimental data. Four are symbolic data and four are numerical data. The datasets are all available at http://mlkd.csd.auth.gr/multilabel.html/#Datasets and http://meka.sourceforge.net/#datasets. Detailed information about the datasets is listed in Table 4. We divided each data set into two parts, eight tenths of which were used as training sets and two as test sets.

First, we examine the sensitivity of the classification effect with respect to the radius of the neighborhood. We run the algorithm at different radii and calculate the corresponding classification metrics. The curves of the classification measures varying with radius are drawn in the figures. The experimental results show that the variation on each dataset is roughly the same. Here, we only list the results for the datasets Scene and Yeast, as shown in Figures 2 and 3.

It can be seen from Figures 2 and 3 that, with the increase of radius, the five classification evaluation measures get better uniformly. At first, the classification effect does not increase significantly and increases sharply when the radius reaches a certain value. However, when the radius increases to a certain extent, the values of the five classification evaluation measures are almost unchanged. On the other hand, corresponding to different parameter *k*, the trend of the curve is basically similar.

From the above analysis, we can conclude that there is an optimal radius for each dataset, and different data correspond to different optimal radius, which does not change with the change of parameter *k*.

In the second experiment, with a given radius, we investigated the sensitivity of the classification accuracy to the parameter *k*. We also draw the curve as shown in Figure 4. We can see that the accuracy curve varies greatly at different radii. When the radius is too small, the parameter *k* does not play any role in the algorithm. For example, the blue curve in Figure 4 when the radius is 0.6. This indicates that the influence of radius on accuracy is more significant than that of parameter *k* in this algorithm. On the other hand, we can roughly conclude from the figures that the accuracy increases with the increase of *k* in the first stage, but decreases when *k* reaches a certain value. Similar to the radius, there is also an optimal parameter *k* for each dataset.

The last pictures in Figures 2, 3, 4, and 5 show the variation of running time with parameters *k* and radius. The running time tends to increase slightly as the two parameters increase, but not significantly. This means that the two parameters have little effect on the speed of the algorithm.

Figure 5 shows the joint effects of two parameters on classification accuracy. When the parameter k is below 10, its influence on classification accuracy is obvious. When the parameter *k* is above 10, the classification accuracy is mainly determined by the radius. We can see the parallel mountains in the graph, their height depends on the radius. This indicates that, relative to parameter *k*, the radius is the determinant of the classification effect. From the point of experiment, it is reasonable to introduce the radius as a parameter in this paper.

In the second part, we compare the operation speeds of five algorithms neighborhood classifier (NC), ML-kNN, BOOSTEXTER, RANK-SVM, and bounded ML-kNN (BML-kNN). Under the same experimental conditions, the algorithms are applied to some generic datasets, and the average running time (s) are shown in Table 5. The underlining indicates the best of the three algorithms.

The experimental results show that the algorithm NC is not advantageous in running time compared with the other algorithms, especially for some datasets with high density. The algorithms ML-kNN and BML-kNN are faster than the other algorithms. However, BML-kNN has a slight numerical advantage, and it performed well on six of the ten datasets, especially on the larger datasets Mediamill and Nus-wide.

In the last part of the experiment, we try to compare the classification accuracy of the three algorithms. At present, the evaluation criteria of multilabel classification in related literature are various. In this paper, we chose five common metrics Hamming loss, One-error, Coverage, Ranking loss, and Average precision. For the definitions and calculation methods, please refer to Reference [1]. Among them, the larger the value of metric Average precision is, the better the classification effect is, and the smaller the value of other measures, the better the classification accuracy. In this paper, we apply the five algorithms to the same datasets and compare the five classification metrics to measure the classification effect of the algorithms.

Tables6–10 show theclassification accuracy under differentmeasures. The numerical values shown in the tables are the average of ten parallel experiments, where the underlines highlight the best over the other algorithms.

As shown in Table 6, from the Hamming loss corresponding to the algorithms, the proposed algorithm BML-kNN has a slight advantage over the other algorithms. However, it is not significant, the numerical difference is the third significant digit in general.

Table 7 reports the experimental results of the classification evaluation One-error. Except the datasets Genbase, Medical, Core15k, and CAL500, BML-kNN works slightly better than the other algorithm. From the experimental results, we can also find that BML-kNN has a prominent performance in all numerical data.

The metric Coverage evaluates the average cost to cover all the true labels. The test results on Coverage are listed in Table 8. The experimental results show that NC and BML-kNN outperform the others. However, the algorithms do not differ much in the numerical value of Coverage. Meanwhile, BML-kNN does not have obvious advantages in the symbol dataset Enron, Medical, Core15k, and Genbase.

Different from other evaluation metrics, the higher the average precision, the better the classification effect. According to the evaluation metrics Average precision and Ranking loss as shown in Tables 9 and 10, BML-kNN is slightly better than NC, and NC is better than the others.

## 5. Conclusions

The proposed algorithm BML-kNN is based on the framework of ML-kNN. ML-kNN only restricts the number of the nearest neighbors, while NC only limits the distance of the nearest neighbors. BML-kNN considers both the two factors at the same time and gives the estimation of test instances based on up to *k* training instances in the neighborhood. Experimental results illustrate that the classification accuracies of BML-kNN and NC are slightly higher than that of ML-kNN. The calculation speeds of BML-kNN and ML-kNN are basically equal, while the algorithm NC has higher computational complexity.

The algorithms involved in this paper divide the multilabel classification problem into a series of single-label problems. Specifically, each label is extracted and combined with the feature data to form a single-label binary classification problem. In this way, the single-label problems are independent of each other, and the correlation between labels is not considered. How to learn the label correlation and apply the correlation into the algorithm may be a meaningful topic for future work.

## Figures and Tables

**Figure 1:** (a) 3NN and (b) bounded 3NN for nonuniformly distributed data.

**Figure 2:** Variation of evaluation metrics with radius of neighborhood on dataset Scene.

**Figure 3:** Variation of evaluation metrics with radius of neighborhood on dataset Yeast.

**Figure 4:** Variation of evaluation metrics with parameter *k* on dataset Yeast.

**Figure 5:** Variation of evaluation metrics with parameter k and radius on dataset Yeast.

**Table 1:** Pseudo-code of ML-kNN.

Input:	*D*, *k*, and unknown instance *t*
Output:	*L*_*t*_
Step 1	For *x* ∈ *X*
Step 2	Identify *k* neighbors *N*^*k*^(*x*)
Step 3	End for
Step 4	For *l* ∈ *L*
Step 5	Learn the probabilities *p*(*C*^*k*^(*x*)=*j*) for *j*=1,2,…, *k*.
Step 8	End for
Step 9	Identify *k* neighbors *N*^*k*^(*t*)
Step 5	For *l* ∈ *L*
Step 6	Calculate the statistics $C^{k}\left(t\right)=\underset{x^{\prime }\in N^{k}\left(t\right)}{\sum }l\left(x^{\prime }\right)$.
Step 8	End for
Step 7	Return *L*_*t*_.

**Table 2:** Pseudo-code of NC.

Input:	*D*, *k*, and unknown instance *t*
Output:	*L*_*t*_
Step 1	For *x* ∈ *X*
Step 2	Identify *k* neighbors *N*_*δ*_(*x*)
Step 3	End for
Step 4	For *l* ∈ *L*
Step 5	Learn the probabilities *p*(*C*_*δ*_(*x*)=*j*) for *j*=1,2,…, *k*.
Step 8	End for
Step 9	Identify *k* neighbors *N*_*δ*_(*t*)
Step 5	For *l* ∈ *L*
Step 6	Calculate the statistics $C_{\delta }\left(t\right)=\underset{x^{\prime }\in N_{\delta }\left(t\right)}{\sum }l\left(x^{\prime }\right)$.
Step 8	End for
Step 7	Return *L*_*t*_.

**Table 3:** Pseudo-code of BML-kNN.

Input:	*X*, *L*, *k*, radius *δ* > 0, and unknown instance *t*
Output:	*l*(*t*), *l* ∈ *L*
Step 1	For *l* ∈ *L*
Step 2	Compute *p*(*l*=1) and *p*(*l*=0) as (13) and (14)
Step 3	$c=\text{zeros}\left(k+1\right),\bar{c}=\text{zeros}\left(k+1\right)$
Step 4	For *x* ∈ *X*
Step 5	Compute *C*(*x*) as (8)
Step 6	If *l*(*x*)==1
Step 7	*c*(*C*(*x*))=*c*(*C*(*x*))+1
Step 8	Else
Step 9	$\bar{c}\left(C\left(x\right)\right)=\bar{c}\left(C\left(x\right)\right)+1$
Step 10	End if
Step 11	End for
Step 12	For *j*=0 : *k*
Step 13	|*D*_*j*_^1^|=*c*(*j*), $\left|D_{j}^{0}\right|=\bar{c}\left(j\right)$
Step 14	Compute *p*(*C*=*j*|*l*=1) and *p*(*C*=*j*|*l*=0) as (17) and (18)
Step 15	End for
Step 16	End for
Step 17	For *l* ∈ *L*
Step 18	Compute *C*(*t*) as (8)
Step 19	Compute *l*(*t*) as (19)
Step 20	End for

**Table 4:** Multilabel data sets.

Dataset	Type	Instances	Features	Label	Domain
Enron	Nominal	1702	1001	53	Text
Medical	Nominal	978	1449	45	Text
Core15k	Nominal	5000	499	374	Images
Genbase	Nominal	662	1185	27	Biology
Yeast	Numerical	2417	103	14	Biology
Emotion	Numerical	593	72	6	Music
CAL500	Numerical	500	62	174	Music
Scene	Numerical	2407	294	6	Images
Mediamill	Numerical	43907	120	101	Video
Nus-wide	Numerical	269648	129	81	Images

**Table 5:** Average running time.

Dataset	ML-kNN	NC	BOOSTEXTER	RANK-SVM	BML-kNN
Yeast	1.73	3.65	1.78	1.88	1.12
Emotion	0.49	0.26	0.33	0.58	0.11
Genbase	0.16	0.33	0.17	0.23	0.19
Scene	1.12	1.35	1.18	1.16	0.61
Enron	0.84	2.52	0.86	0.89	0.97
Medical	0.34	0.82	0.62	0.78	0.39
Core15k	12.1	46.4	18.2	19.2	15.8
CAL500	1.53	1.87	1.49	1.64	1.43
Mediamill	82.1	90.7	87.0	81.1	76.6
Nus-wide	565	596	529	581	547

**Table 6:** Hamming loss.

Dataset	ML-kNN	NC	BOOSTEXTER	RANK-SVM	BML-kNN
Yeast	0.22	0.26	0.28	0.27	0.21
Emotion	0.27	0.29	0.26	0.24	0.23
Genbase	0.04	0.07	0.05	0.06	0.03
Scene	0.09	0.09	0.11	0.07	0.10
Enron	0.06	0.07	0.08	0.07	0.05
Medical	0.01	0.02	0.03	0.03	0.02
Core15k	0.01	0.02	0.02	0.02	0.02
CAL500	0.11	0.13	0.12	0.12	0.09
Mediamill	0.03	0.04	0.05	0.04	0.02
Nus-wide	0.02	0.02	0.03	0.02	0.01

**Table 7:** One-error.

Dataset	ML-kNN	NC	BOOSTEXTER	RANK-SVM	BML-kNN
Yeast	0.25	0.29	0.26	0.28	0.22
Emotion	0.38	0.39	0.36	0.37	0.35
Genbase	0.02	0.02	0.03	0.01	0.02
Scene	0.24	0.31	0.27	0.28	0.22
Enron	0.31	0.34	0.38	0.41	0.39
Medical	0.27	0.28	0.31	0.28	0.26
Core15k	0.74	0.73	0.79	0.76	0.80
CAL500	0.12	0.15	0.17	0.12	0.11
Mediamill	0.17	0.19	0.20	0.18	0.16
Nus-wide	0.57	0.60	0.67	0.58	0.56

**Table 8:** Coverage.

Dataset	ML-kNN	NC	BOOSTEXTER	RANK-SVM	BML-kNN
Yeast	6.22	6.31	6.25	6.27	6.16
Emotion	2.31	2.36	2.33	2.37	2.29
Genbase	0.56	0.53	0.56	0.61	0.59
Scene	0.45	0.47	0.49	0.50	0.44
Enron	15.4	15.1	14.4	14.1	13.9
Medical	2.49	2.45	2.61	2.56	2.64
Core15k	115	112	121	113	122
CAL500	113	117	126	123	126
Mediamill	19.0	20.1	20.2	19.6	18.9
Nus-wide	14.0	13.6	13.9	13.8	13.3

**Table 9:** Average precision.

Dataset	ML-kNN	NC	BOOSTEXTER	RANK-SVM	BML-kNN
Yeast	0.78	0.73	0.77	0.83	0.87
Emotion	0.62	0.67	0.65	0.69	0.71
Genbase	0.98	0.98	0.97	0.98	0.99
Scene	0.89	0.86	0.83	0.82	0.86
Enron	0.63	0.59	0.62	0.61	0.65
Medical	0.80	0.89	0.83	0.85	0.87
Core15k	0.23	0.21	0.20	0.24	0.19
CAL500	0.46	0.43	0.45	0.47	0.49
Mediamill	0.69	0.67	0.66	0.69	0.72
Nus-wide	0.46	0.47	0.49	0.51	0.52

**Table 10:** Ranking loss.

Dataset	ML-kNN	NC	BOOSTEXTER	RANK-SVM	BML-kNN
Yeast	0.18	0.19	0.23	0.21	0.25
Emotion	0.25	0.23	0.22	0.23	0.26
Genbase	0.02	0.01	0.03	0.02	0.02
Scene	0.09	0.14	0.11	0.13	0.07
Enron	0.10	0.12	0.13	0.09	0.12
Medical	0.05	0.1297	0.19	0.19	0.14
Core15k	0.14	0.13	0.12	0.17	0.14
CAL500	0.18	0.18	0.19	0.19	0.17
Mediamill	0.06	0.07	0.09	0.08	0.05
Nus-wide	0.12	0.14	0.13	0.12	0.11

## Data Availability

The data used to support the findings of this study are included within the article.
